RETRACTED

# Guanylate‐binding protein 1 correlates with advanced tumor features, and serves as a prognostic biomarker for worse survival in lung adenocarcinoma patients

**DOI:** 10.1002/jcla.23610

**Published:** 2020-12-10

**Authors:** Quanchao Wan, Jingming Qu, Longfei Li, Feng Gao

**Affiliations:** ^1^ Department of Cardiothoracic Surgery Xuzhou Cancer Hospital Xuzhou China

**Keywords:** guanylate‐binding protein 1, immunohistochemistry assay, lung adenocarcinoma, survival, tumor features

## Abstract

**Objective:**

Guanylate‐binding protein 1 (GBP1) is reported to promote tumor progression and treatment resistance in lung cancer, and presents as a prognostic biomarker in several solid tumors. However, the related research of GBP1 in clinical management of lung adenocarcinoma is still lacking. Therefore, the present study aimed to detect the clinical role of GBP1 in lung adenocarcinoma.

**Methods:**

The clinical data of 221 lung adenocarcinoma patients were retrospectively analyzed, and then, their tumor tissue specimens and paired adjacent tissue specimens were retrieved for GBP1 detection via immunohistochemistry (IHC) assay.

**Results:**

GBP1 expression was upregulated in tumor tissues compared with adjacent tissues (*P* < .001). Moreover, high tumor GBP1 expression was associated with larger tumor size (*P* = .030), positive lymph node (LYN) metastasis (*P* = .001), advanced TNM stage (*P* = .001), and abnormal preoperative carcinoembryonic antigen (CEA) level (*P* = .026). Furthermore, tumor GBP1 high expression was correlated with reduced disease‐free survival (DFS) and overall survival (OS), and was of independent value in predicting worse DFS and OS. Additionally, data analysis of 1144 lung cancer patients derived from KMplot database (www.kmplot.com) further verified that GBP1 expression was negatively correlated with OS (*P* = .009).

**Conclusion:**

GBP1 correlates with advanced tumor features and worse survival profiles, suggesting its value to be a prognostic biomarker in management of lung adenocarcinoma.

## Graphical abstract

**Methods:** The clinical data of 221 lung adenocarcinoma patients were retrospectively analyzed, and then, their tumor tissue specimens and paired adjacent tissue specimens were retrieved for GBP1 detection via immunohistochemistry (IHC) assay. According to total GBP1 IHC stain scoring in specimens, the score ≤3 was defined as GBP1 low expression, while the score >3 was defined as GBP1 high expression.

## 1 INTRODUCTION

Lung cancer remains the leading contributor to cancer incidence, and represents approximately 20% cancer‐related deaths globally.^1^, ^2^ Lung adenocarcinoma is the most common subtype of lung cancer, and includes adenocarcinoma in situ (AIS), minimally invasive adenocarcinoma (MIA), and invasive adenocarcinomas.^3^ Despite the achievements in pathogenesis understanding and treatment advancements of lung adenocarcinoma, such as the development of individualized therapies, lung adenocarcinoma is still a devastating and aggressive tumor type considering the high risk of distant metastasis and acquired treatment resistance.^3^, ^4^ Therefore, it is essential to explore the underlying mechanism of lung adenocarcinoma and look for novel prognostic biomarkers, assisting the management of lung adenocarcinoma.

RETRACTED

Guanylate‐binding protein 1 (GBP1) is a GTP‐binding protein with a high GTPase activity, which interacts with various binding proteins involving in diverse biological functions, such as extracellular signaling, endosomal trafficking, and signal transduction.^5^ As for at cellular level, GBP1 serves as a cellular mediator of interferon‐gamma (IFN‐γ) and is implicated in diverse IFN‐γ–mediated cellular responses in various cell lines, including bronchial epithelial cells.^5^, ^6^, ^7^ Furthermore, the role of GBP1 has been demonstrated in several lung‐related diseases, which reveal that GBP1 is aberrantly expressed in patients with acute respiratory distress syndrome and pulmonary sarcoidosis.^8^, ^9^ In addition, given that cancer emerges from a complex interaction between mutational events and cell state transitions accompanying by IFN‐mediated inflammation, GBP1 is reported to participate in the oncogenic process of lung cancer.^10^, ^11^, ^12^ For example, GBP1 promotes tumor progression and paclitaxel resistance via activating Wnt/β‐catenin signaling pathway in non–small‐cell lung cancer (NSCLC).^10^ In addition, one study indicates that GBP1 promotes cell migration and invasion in lung adenocarcinoma.^12^ According to aforementioned evidence, we hypothesized that GBP1 might have potential to be a clinical prognostic biomarker of lung adenocarcinoma; however, there was no related study. Herein, we determined the expression of GBP1 in patients with lung adenocarcinoma, and further analyzed the correlation of GBP1 with clinical characteristics and prognosis of lung adenocarcinoma.

## 2 MATERIALS AND METHODS

### 2.1 Patients

This study retrospectively analyzed 221 patients with lung adenocarcinoma who underwent surgical resection in our hospital between January 2012 and December 2014. All analyzed patients met following criteria: (a) pathologically diagnosed as primary lung cancer; (b) histologically confirmed as lung adenocarcinoma; (c) age more than 18 years; (d) had well‐preserved tumor and adjacent tissue specimens that were removed during the surgery; and (e) had complete preoperative clinical data and follow‐up records that were able to use for assessment of disease‐free survival (DFS) and OS. Patients who received neoadjuvant therapy before surgery, complicated with other cancers or without any follow‐up data, were not included in the study. After surgery, patients received appropriate adjuvant therapy if clinically indicated (eg, chemotherapy and radiation therapy), according to NCCN guideline of NSCLC (NCCN: Non‐Small Cell Lung Cancer Version 1.2013.).^13^ The approval by Institutional Review Board of our hospital was obtained before initiation of study. The written informed consents were collected from patients or their family members.

RETRACTED

### 2.2 Data collection

Preoperative clinical data of patients were collected from the medical records, which covered age, gender, history of smoke, history of drink, hypertension, hyperlipidemia, diabetes, tumor differentiation, tumor size, lymph node (LYN) metastasis, TNM stage, and carcinoembryonic antigen (CEA) level. In addition, patients were followed up by clinic visits or telephone calls every 3‐6 months. The survival data of patients were collected from follow‐up records, which included disease status, disease relapse date, survival status, death date of patients, and last visit date. According to the survival data, DFS was calculated from the date of surgery to the date of disease relapse or patients’ death; OS was calculated from the date of surgery to the date of patients’ death or last visit. Patients who did not suffer from disease relapse or death were censored on the date of last visit in the survival analysis.

### 2.3 Immunohistochemistry (IHC) assay

Totally 221 formaldehyde fixed, paraffin‐embedded (FFPE) tumor tissue specimens and paired adjacent tissue specimens were collected from pathology department of our hospital. GBP1 expression in FFPE specimens was determined by IHC assay. Briefly, FFPE specimens were cut into 4‐μm slices, mounted on positively charged glass slides and air‐dried overnight. Next, the slices were deparaffinized in xylene and rehydrated in ethanol, then were quenched with fresh hydrogen peroxide to inhibit endogenous tissue peroxidase activity. After that, the slices were placed in antigen retrieval buffer and brought up to boil. Subsequently, slices were incubated with GBP1 polyclonal antibody (Thermo Fisher Scientific) at 4°C overnight. Next day, the slices were incubated with goat anti‐rabbit IgG (H + L) secondary antibody (Thermo Fisher Scientific) at room temperature for 30 minutes. Afterward, slices were stained with diaminobenzidine and counterstained with hematoxylin. The slices were finally evaluated by investigator under a light microscopy.

RETRACTED

### 2.4 GBP1 expression evaluation

Based on the staining intensity and positively stained cell density, the GBP1 expression in the specimens was evaluated using a semi‐quantitative scoring method as described in a previous study.^14^ The staining intensity was scored as 0, negative; 1, weak; 2, moderate; and 3, strong. The positively stained cell density was represented by percentage of positively stained cells, which was scored as: 0, 0%; 1, 1%‐25%; 2, 26%‐50%; 3, 51%‐75%; and 4, 76%‐100%. After multiplying the staining intensity score by the positively stained cell density score, a total IHC staining score of each specimen was obtained, which was ranging from 0 to 12. The total IHC staining score ≤3 was defined as GBP1 low expression; accordingly, total IHC staining score >3 was defined as GBP1 high expression.^14^

### 2.5 Derived data of association between GBP1 and OS from KMplot database (www.kmplot.com)

We further verified the association between GBP1 and OS in 1144 lung cancer patients derived from an integrated database (KMplot, www.kmplot.com) of previously published transcriptomic datasets. The integrated database was developed as an online tool suitable for the real‐time meta‐analysis of published lung cancer microarray datasets to identify biomarkers related to survival,^15^ where univariate and multivariate Cox regression analysis, Kaplan‐Meier survival plot with hazard ratio, and log‐rank P value were calculated and plotted in R. The complete analysis tool could be accessed online at: www.kmplot.com/lung.

### 2.6 Statistical analysis

All data analyses were carried out using SPSS 22.0 statistical software (IBM), and all graphs were plotted using GraphPad Prism 7.01 (GraphPad Software Inc). Clinical data were described as mean with standard deviation (SD), median with interquartile range (IQR), or number with percentage (No. (%)). GBP1 expression difference between tumor tissue and adjacent tissue was determined by McNemar's test. Correlation of tumor GBP1 with clinical features of patients was determined by the chi‐square test or the Spearman rank correlation test. Association between tumor GBP1 and DFS/OS was determined by log‐rank test, which was displayed by the Kaplan‐Meier curve. DFS‐related factors and OS‐related factors were identified by univariate and forward stepwise multivariate Cox's proportional hazards regression analyses. Statistical significance level was defined as *P* value < .05.

## 3 RESULTS

### 3.1 Clinical characteristics in patients with lung adenocarcinoma

The mean age of patients was 61.5 ± 10.8 years (Table 1). The number of male and female patients was 172 (77.8%) and 49 (22.2%), respectively. There were 32 (14.5%), 128 (57.9%), and 61 (27.6%) patients with well, moderate, and poor pathological differentiation, respectively. The average tumor size was 5.2 ± 2.1 cm. The number of patients with positive LYN metastasis was 79 (35.7%). As for TNM stage, the number of patients with TNM stages I, II, and III was 79 (35.7%), 59 (26.7%), and 83 (37.6%), respectively. The number of patients with abnormal preoperative CEA level (>5 ng/mL) was 132 (59.7%). The detailed information of clinical characteristics in patients with lung adenocarcinoma is shown in Table 1.

RETRACTED

**TABLE 1:** Clinical features of patients with lung adenocarcinoma

Items	Patients (N = 221)
Age (y), mean ± SD	61.5 ± 10.8
≤60 y, No. (%)	109 (49.3)
>60 y, No. (%)	112 (50.7)
Gender, No. (%)	
Male	172 (77.8)
Female	49 (22.2)
History of smoke, No. (%)	112 (50.7)
History of drink, No. (%)	82 (37.1)
Comorbidities, No. (%)	
Hypertension	80 (36.2)
Hyperlipidemia	64 (29.0)
Diabetes	30 (13.6)
Pathological differentiation, No. (%)	
Well	32 (14.5)
Moderate	128 (57.9)
Poor	61 (27.6)
Tumor size (cm), mean ± SD	5.2 ± 2.1
≤5 cm	136 (61.5)
>5 cm	85 (38.5)
LYN metastasis, No. (%)	
Negative	142 (64.3)
Positive	79 (35.7)
TNM stage, No. (%)	
Stage I	79 (35.7)
Stage II	59 (26.7)
Stage III	83 (37.6)
Preoperative CEA level (ng/mL), median (IQR)	
Normal (≤5 ng/mL)	89 (40.3)
Abnormal (>5 ng/mL)	132 (59.7)

Abbreviations: CEA, carcinoembryonic antigen; IQR, interquartile range; LYN, lymph node; SD, standard deviation.

### 3.2 Comparison of GBP1 expression between tumor and adjacent tissues in lung adenocarcinoma patients

After multiplying the staining intensity score by the positively stained cell density score, the total IHC staining score was ranging from 0 to 12. The total IHC staining score ≤3 was defined as GBP1 low expression, and total IHC staining score >3 was defined as GBP1 high expression. The representative example of GBP1 low and high expression in adjacent and tumor tissues is shown in Figure 1. Further comparative analysis indicated that, in tumor tissue, the proportion of GBP1 low expression and high expression were 51.6% and 48.4%, respectively; as for in adjacent tissue, the proportion of GBP1 low expression and high expression were 69.7% and 30.3%, respectively (Table 2). It is important that GBP1 expression was upregulated in tumor tissue compared with adjacent tissue (*P* < .001).

**FIGURE 1:** Representative images of GBP1 IHC expression in tumor and adjacent tissue. After multiplying the staining intensity score by the positively stained cell density score, a total IHC staining score of each specimen was obtained, which was ranging from 0 to 12, and the score ≤3 was defined as GBP1 low expression, while the score >3 was defined as GBP1 high expression. GBP1, guanylate‐binding protein 1; IHC, immunohistochemistry

**TABLE 2:** GBP1 expression in tumor and adjacent tissue

	GBP1 expression		*P* value
	Low	High	
Tumor tissue (N = 221)	114 (51.6)	107 (48.4)	<.001
Adjacent tissue (N = 221)	154 (69.7)	67 (30.3)	

Abbreviation: GBP1, guanylate‐binding protein 1.

RETRACTED

### 3.3 Correlation of tumor GBP1 expression with clinical characteristics in lung adenocarcinoma patients

High tumor GBP1 expression was associated with larger tumor size (*P* = .030), positive LYN metastasis (*P* = .001), advanced TNM stage (*P* = .001), and abnormal preoperative CEA level (>5 ng/mL) (*P* = .026) (Table 3). However, there was no correlation of tumor GBP1 expression with age, gender, history of smoke, history of drink, hypertension, hyperlipidemia, diabetes, or pathological differentiation (all *P* > .05). The detailed information of clinical characteristics between tumor GBP1 high patients and tumor GBP1 low patients is displayed in Table 3.

**TABLE 3:** Correlation of tumor GBP1 expression with clinical features

Items	Tumor GBP1 expression		*P* value
	Low (n = 114)	High (n = 107)	
Age, No. (%)			
≤60 y	55 (48.2)	54 (50.5)	.741
>60 y	59 (51.8)	53 (49.5)	
Gender, No. (%)			
Male	91 (79.8)	81 (75.7)	.461
Female	23 (20.2)	26 (24.3)	
History of smoke, No. (%)			
No	52 (45.6)	57 (53.3)	.255
Yes	62 (54.4)	50 (46.7)	
History of drink, No. (%)			
No	76 (66.7)	63 (58.9)	.231
Yes	38 (33.3)	44 (41.1)	
Hypertension, No. (%)			
No	69 (60.5)	72 (67.3)	.296
Yes	45 (39.5)	35 (32.7)	
Hyperlipidemia, No. (%)			
No	77 (67.5)	80 (74.8)	.237
Yes	37 (32.5)	27 (25.2)	
Diabetes, No. (%)			
No	100 (87.7)	91 (85.0)	.562
Yes	14 (12.3)	16 (15.0)	
Pathological differentiation, No. (%)			
Well	18 (15.8)	14 (13.1)	.698
Moderate	65 (57.0)	63 (58.9)	
Poor	31 (27.2)	30 (28.0)	
Tumor size, No. (%)			
≤5 cm	78 (68.4)	58 (54.2)	.030
>5 cm	36 (31.6)	49 (45.8)	
LYN metastasis, No. (%)			
Negative	85 (74.6)	57 (53.3)	.001
Positive	29 (25.4)	50 (46.7)	
TNM stage, No. (%)			
Stage I	52 (45.6)	27 (25.2)	.001
Stage II	29 (25.4)	30 (28.0)	
Stage III	33 (28.9)	50 (46.8)	
Preoperative CEA level, No. (%)			
Normal (≤5 ng/mL)	54 (47.4)	35 (32.7)	.026
Abnormal (>5 ng/mL)	60 (52.6)	72 (67.3)	

Abbreviations: CEA, carcinoembryonic antigen; GBP1, Guanylate‐binding protein 1; LYN, lymph node.

### 3.4 Correlation of tumor GBP1 expression with disease relapse and survival in lung adenocarcinoma patients

Further analysis compared the survival profiles between tumor GBP1 high patients and tumor GBP1 low patients, which observed that tumor GBP1 high expression was correlated with decreased DFS (*P* < .001) (Figure 2A) and OS (*P* < .001) (Figure 2B) in lung adenocarcinoma patients. Furthermore, the correlation of GBP1 with OS was further verified by the data of 1144 lung cancer patients derived from KMplot database (www.kmplot.com), which observed that OS was decreased in patients with GBP1 high expression compared to those with GBP1 low expression (*P* = .009) (Figure 3). However, this database was based on mRNA sequencing, which could not verify the correlation of GBP1 protein expression with OS.

RETRACTED

**FIGURE 2:** Correlation of GBP1 with survival profiles. Correlation of GBP1 with DFS (A) and OS (B) in lung adenocarcinoma patients recruited. GBP1, guanylate‐binding protein 1; DFS, disease‐free survival; OS, overall survival

**FIGURE 3:** Data from KMplot database. Correlation of GBP1 mRNA level with OS in 1144 lung cancer patients derived from KMplot database (KMplot, www.kmplot.com). GBP1, guanylate‐binding protein 1; OS, overall survival

### 3.5 Factors affecting DFS in lung adenocarcinoma patients

To further detect the correlation of GBP1 expression with DFS in lung adenocarcinoma patients, we conducted univariate Cox's proportional hazard regression and found that GBP1 high expression (HR = 1.828, *P* < .001), worse pathological differentiation (HR = 1.277, *P* = .033), tumor size >5 cm (HR = 1.458, *P* = .014), LYN metastasis positive (HR = 2.805, *P* < .001), higher TNM stage (HR = 1.477, *P* < .001), and preoperative CEA abnormal (>5 ng/mL) (HR = 1.526, *P* = .007) were correlated with worse DFS (Table 4). Further multivariate Cox's proportional hazard regression revealed that GBP1 high expression (HR = 1.537, *P* = .004), LYN metastasis positive (HR = 2.495, *P* < .001), and preoperative CEA abnormal (>5 ng/mL) (HR = 1.409, *P* = .029) were independent factors for reduced DFS.

**TABLE 4:** DFS‐related factors

Items	Cox's proportional hazard regression	
	HR (95% CI)	*P* value
Univariate Cox's regression		
GBP1 high expression	1.829 (1.357‐2.465)	<.001
Age >60 y	1.178 (0.876‐1.586)	.278
Male	1.109 (0.769‐1.600)	.578
History of smoke	0.940 (0.700‐1.262)	.680
History of drink	1.214 (0.897‐1.642)	.209
Hypertension	1.051 (0.772‐1.432)	.751
Hyperlipidemia	1.111 (0.801‐1.539)	.529
Diabetes	1.305 (0.860‐1.980)	.211
Worse pathological differentiation	1.277 (1.020‐1.598)	.033
Tumor size >5 cm	1.458 (1.079‐1.970)	.014
LYN metastasis positive	2.805 (2.063‐3.816)	<.001
Higher TNM stage	1.477 (1.237‐1.763)	<.001
Preoperative CEA abnormal (>5 ng/mL)	1.526 (1.125‐2.070)	.007
Multivariate Cox's regression (forward stepwise)		
GBP1 high expression	1.573 (1.159‐2.134)	.004
LYN metastasis positive	2.495 (1.822‐3.415)	<.001
Preoperative CEA abnormal (>5 ng/mL)	1.409 (1.036‐1.915)	.029

Abbreviations: CEA, carcinoembryonic antigen; CI, confidence interval; DFS, disease‐free survival; GBP1, Guanylate‐binding protein 1; HR, hazard ratio; LYN, lymph node.

RETRACTED

### 3.6 Factors affecting OS in lung adenocarcinoma patients

To further detect the correlation of GBP1 expression with OS in lung adenocarcinoma patients, univariate Cox's proportional hazard regression was performed, which observed that GBP1 high expression (HR = 2.218, *P* < .001), worse pathological differentiation (HR = 1.367, *P* = .013), tumor size >5 cm (HR = 1.620, *P* = .004), LYN metastasis positive (HR = 3.506, *P* < .001), higher TNM stage (HR = 1.430, *P* < .001), and preoperative CEA abnormal (>5 ng/mL) (HR = 2.058, *P* < .001) were correlated with decreased OS (Table 5). Further multivariate Cox's proportional hazard regression revealed that GBP1 high expression (HR = 1.756, *P* = .001), worse pathological differentiation (HR = 1.301, *P* = .044), LYN metastasis positive (HR = 3.023, *P* < .001), and preoperative CEA abnormal (>5 ng/mL) (HR = 1.917, *P* < .001) were independent factors for decreased OS.

**TABLE 5:** OS‐related factors

Items	Cox's proportional hazard regression	
	HR (95% CI)	*P* value
Univariate Cox's regression		
GBP1 high expression	2.218 (1.591‐3.093)	<.001
Age >60 years	1.077 (0.779‐1.490)	.652
Male	0.907 (0.618‐1.332)	.620
History of smoke	1.015 (0.735‐1.404)	.926
History of drink	1.172 (0.841‐1.634)	.348
Hypertension	1.166 (0.834‐1.631)	.369
Hyperlipidemia	1.163 (0.817‐1.656)	.403
Diabetes	1.322 (0.840‐2.081)	.228
Worse pathological differentiation	1.367 (1.068‐1.749)	.013
Tumor size >5 cm	1.620 (1.169‐2.245)	.004
LYN metastasis positive	3.506 (2.515‐4.888)	<.001
Higher TNM stage	1.430 (1.179‐1.736)	<.001
Preoperative CEA abnormal (>5 ng/mL)	2.058 (1.451‐2.920)	<.001
Multivariate Cox's regression (forward stepwise)		
GBP1 high expression	1.756 (1.249‐2.470)	.001
Worse pathological differentiation	1.301 (1.007‐1.681)	.044
LYN metastasis positive	3.023 (2.156‐4.241)	<.001
Preoperative CEA abnormal (>5 ng/mL)	1.917 (1.348‐2.724)	<.001

Abbreviations: CEA, carcinoembryonic antigen; CI, confidence interval; GBP1, guanylate‐binding protein 1; HR, hazard ratio; LYN, lymph node; OS, overall survival.

## 4 DISCUSSION

GBP1 is an important member of the GTPase family, and its structure consists of two domains, including a N‐terminal globular domain with GTPase activity and a C‐terminal α‐helical domain.^16^ Several recent studies reveal the involvement of GBP1 in the underlying mechanism of different tumors, such as prostate cancer, ESCC, and ovarian cancer.^11^, ^17^, ^18^ For example, mechanically, GBP1 promotes cell proliferation, migration, and invasion, and increases the level of mitochondrial oxidative phosphorylation and glycolysis in prostate cancer cells, enhancing progression and aggression of prostate tumor.^11^ Further clinical correlation analysis exhibits that GBP1 is correlated with aggressive clinical features and shorter survival profiles in prostate cancer patients.^11^ In addition, the implication of GBP1 in lung cancer is indicated by previous publication, which reports that GBP1 enhances cell motility to promote lung adenocarcinoma invasiveness.^12^ However, the correlation of GBP1 with clinical characteristics and prognosis is not determined in lung adenocarcinoma patients yet, which was explored in our present study.

RETRACTED

In our present study, we detected GBP1 expression in tumor and pair adjacent tissues of lung adenocarcinoma patients via IHC assay and found that GBP1 was upregulated in lung adenocarcinoma tissues compared with paired adjacent tissues. The possible reasons might include that (a) according to previous studies, GBP1 might have pro‐survival effects on some oncogenic mutations, such as EGFR mutation, leading to EGFR mutation‐driven tumorigenicity of lung adenocarcinoma^19^; and (b) in addition, GBP1 might exert oncogenic effect and its high expression might activate oncogenic Wnt/β‐catenin signaling pathway, contributing to the initiation of lung adenocarcinoma.^10^

Furthermore, we further detected the correlation of GBP1 with clinical characteristics in lung adenocarcinoma patients, and found that its high expression was correlated with larger tumor size, presence of LYN metastasis, advanced TNM stage, and abnormal preoperative CEA level, suggesting the positive correlation of GBP1 with advanced tumor features of lung adenocarcinoma. The possible reasons might include that (a) based on the correlation of GBP1 with EGFR mutation, GBP1 might lead to autophosphorylation of receptor tyrosine kinase via activating EGFR, initiating a cascade of downstream signaling pathway, and further resulting in cellular proliferation, differentiation, and survival of lung adenocarcinoma. Therefore, high GBP1 expression was correlated with development and progression of lung adenocarcinoma^20^; and (b) in addition, GBP1 was reported to be involved in the actin cytoskeleton remodeling process that was an essential event in cell migration, and therefore, we speculated that GBP1 high expression might promote cell motility and invasiveness of lung adenocarcinoma, and further correlate with LYN metastasis and advanced TNM stage in lung adenocarcinoma patients.^21^

Previous evidence has indicated the correlation of GBP1 with the development of treatment resistance.^10^, ^11^, ^22^ For example, GBP1 is correlated with ovarian tumor recurrence after paclitaxel or docetaxel therapies, and its high expression predicts a significantly decreased progression‐free survival in ovarian cancer patients.^10^ As for in NSCLC, another experimental study reveals that drug resistance to paclitaxel is reversed after the GBP1 knockdown in NSCLC cells with paclitaxel resistance..^22^ In addition, considering the correlation of GBP1 with advanced tumor features in lung adenocarcinoma patients and given the correlation of GBP1 with therapy resistance in tumor treatment, further analysis was conducted to explore the association of GBP1 with survival profiles in the patients recruited in the present study.^10^, ^11^, ^22^ The results observed that GBP1 was negatively correlated with reduced DFS and OS, and was of independent value in predicting worse DFS and OS in lung adenocarcinoma patients. This result was further validated by the data derived from KMplot database, and these results both suggested that GBP1 presented value to be a prognostic biomarker in lung adenocarcinoma. The possible reasons might involve that (a) firstly, according to prior results, GBP1 high expression was associated with advanced tumor features in lung adenocarcinoma patients, which were considered to be high risk factors for poor prognosis. Therefore, lung adenocarcinoma patients with higher GBP1 expression presented with poor survival^23^; (b) secondly, GBP1 might promote the invasiveness of lung adenocarcinoma via promoting cell motility, increasing the recurrence risk and contributing to undesirable survival profiles in patients with lung adenocarcinoma^12^; (c) thirdly, considering the correlation of GBP1 with increased chemotherapy resistance, patients with GBP1 high expression might present reduced treatment response, and further long‐term worse survival profiles.^11^, ^22^ Furthermore, as the current study was a single‐center study with a relatively small sample size, there therefore might exist sampling bias and limited generalization, which contributed to more significant in the study samples compared with that extracted from KMplot database.

RETRACTED

There still existed some limitations in present study as follows: (a) Firstly, the present study was a single‐center study with a relatively small sample size; therefore, further studies recruiting more patients from multiple centers were needed for validation. (b) Secondly, the detailed mechanism of GBP1 involving in molecular pathways driving tumor progression and its contribution to treatment resistance in lung adenocarcinoma needed further cellular experiments for investigation. (c) Thirdly, our study only detected the protein expression of GBP1 by IHC assay, and more detection techniques (such as reverse transcription quantitative polymerase chain reaction used for GBP1 mRNA quantification) were needed to further validating the results. (d) Fourthly, the present study only included the patients with lung adenocarcinoma; therefore, the value of GBP1 as a prognostic biomarker in the management of lung squamous cell carcinoma needed further exploration. (e) Fifthly, the median of follow‐up duration was 56 months (range: 2 months‐96 months), and longer follow‐up period was needed for further validating the long‐term clinical role of GBP1 in the management of lung adenocarcinoma.

In conclusion, GBP1 is correlated with advanced tumor features, unfavorable DFS, and OS, suggesting its potential as a prognostic biomarker in management of lung adenocarcinoma.
